# Clinical Curative Effects and Influencing Factors of Uterine Artery Chemoembolization Combined with Uterine Curettage Treating with Cesarean Scar Pregnancy Patients

**DOI:** 10.1155/2022/7785573

**Published:** 2022-09-27

**Authors:** Kewen Yu, Haifeng Zhou

**Affiliations:** ^1^Department of Gynecology, Ningbo Women and Children's Hospital, Ningbo 315010, Zhejiang, China; ^2^Department of Obsterics and Gynecology, Zhuji Maternal and Child Health Hospital, Zhuji 311800, Zhejiang, China

## Abstract

**Objective:**

To explore the clinical curative effects of uterine arterial chemoembolization (UACE) combined with uterine curettage treating with cesarean scar pregnancy (CSP) patients, and analyze the influencing factors of postoperative efficacy.

**Methods:**

A total of 86 patients with CSP from January 2019 to December 2021 in the Gynecology ward of our hospital were selected and divided into the control group (*n* = 43) and the observation group (*n* = 43) according to the random number method. The control group was treated with an injection of methotrexate (MTX) combined with uterine curettage, and the observation group was treated with UACE combined with uterine curettage. Two months after the operation, the therapeutic effect, cesarean scar mass, and *β*-human chorionic gonadotropin (*β*-HCG) level were observed and compared between the two groups. The general conditions of patients in two groups were recorded, and the influencing factors of surgical efficacy in patients were analyzed using univariate analysis and a multivariate logistic regression model.

**Results:**

After treatment, the total effective rate of the observation group was significantly higher than that of the control group (*P* < 0.05). The volume of intraoperative blood loss, hospitalization period, menstrual recovery time, mass disappearance time, and *β*-HCG recovery time of the observation group were lower than those of the control group (*P* < 0.05). Single factor analysis showed that the number of cesarean sections, gestational age, the largest diameter of the gestational sac, the thinnest muscular layer, and the type of CSP can all affect postoperative efficacy (*P* < 0.05). Multivariate logistic analysis showed that the gestational age, a maximum diameter of a gestational sac, the thinnest muscular layer, and the type of CSP were independent factors influencing the postoperative efficacy of the patients (*P* < 0.05).

**Conclusion:**

UACE combined with uterine curettage for CSP can significantly improve the curative effect, reduce intraoperative bleeding, and improve the recovery time of postoperative-related symptoms. The gestational age of the patient, the maximum diameter of the gestational sac, the thinnest muscular layer, and the type of CSP can independently affect the therapeutic effect of CSP patients. Fully understanding the high-risk factors that affect the efficacy of treatment of CSP, timely preventive measures, and targeted care can effectively improve the prognosis and reduce the risk of CSP.

## 1. Introduction

Cesarean scar pregnancy (CSP) refers to the growth and development of fertilized eggs in the scar of a previous cesarean section, which belongs to a special kind of ectopic pregnancy. With the opening of the second child and the maturity of cesarean section in China, the incidence of CSP is increasing year by year [1, 2]. Currently, the incidence of CSP accounts for about 0.5% of the total number of pregnancies. Because the myometrium of cesarean section scar is weak and the blood supply is rich, if the diagnosis and treatment of cesarean section scar pregnancy cannot be made in time, the patient will have the risk of uterine rupture and massive hemorrhage, which will seriously endanger the life of the patient [3, 4]. Currently, the methods of treating cesarean scar pregnancy include total hysterectomy, methotrexate (MTX) combined with uterine clearance, and uterine artery chemoembolization (UACE) combined with uterine clearance. [5]. Among many methods, UACE is an interventional therapy that injects an embolic agent into a blood vessel under ultrasound, CT, or X-ray guidance to reduce massive hemorrhage in a patient [6, 7]. This study investigated the efficacy of UACE combined with uterine curettage in the treatment of cesarean scar pregnancy, and the related factors affecting the efficacy. The specific report is as follows.

## 2. Materials and Methods

### 2.1. General Information

The clinical data of 86 patients with cesarean section scar pregnancy who were hospitalized in the gynecological ward of our hospital from January 2019 to December 2021 were retrospectively collected. They were divided into the control group and the observation group by random number method, with 43 cases in each group. In the control group, the age was 20–35 years old, with an average of (26.95 ± 3.42) years old; 2^nd^ pregnancy times (1∼4); 26 cases of CSP Type 1 and 17 cases of CSP Type 2. In the observation group, the age was 19–36 years old, with an average of (27.25 ± 4.01) years old; 2^nd^ pregnancy times (1∼3); 24 cases of CSP Type 1 and 19 cases of CSP Type 2. There was no statistically significant difference in general data such as age and pregnancy between the two groups, and they were comparable (*P* > 0.05).

### 2.2. Inclusion and Exclusion Criteria

#### 2.2.1. Inclusion Criteria

Inclusion criteria were as follows: patients who meet the diagnostic criteria of CSP (the ultrasonic diagnosis showed that there was no fetal sac in the normal position of the uterine cavity, and the fetal sac appeared in the lower part of the uterine cavity, and the fetal sac locally protruded to the cesarean section scar site, or it was directly located in the cesarean section scar diverticulum) [8]; under the age of 40; patients with type I or type II CSP (both diagnosed and classified by a gynecologic three-dimensional ultrasound performed by an experienced sonographer); patients with serum *β*-human chorionic gonadotropin (*β*-HCG) ≥ 10000 mIU/mL; the vital signs are stable; the liver and kidney function and coagulation function are normal; and no history of allergy to iodinated contrast media and methotrexate.

#### 2.2.2. Exclusion Criteria

Exclusion criteria were as follows: patients with type III CSP or type I CSP with a course of less than 8 weeks; Patients with serum *β*-HCG < 10000 mIU/ml; patients with vaginal bleeding, unstable vital signs, or shock before treatment; or patients with severe liver and kidney function and coagulation function; Patients with contraindications for UACE.

### 2.3. Research Methods

The control group was treated with MTX combined with ultrasound-guided uterine curettage. Perform ultrasound-guided intravaginal or intra-abdominal injection of MTX, 50 mg/m^2^ each time, and review the blood *β*-HCG after 5 days. If the increase or decrease of this index is less than 15%, MTX 50 mg/m^2^ is injected again on the 6^th^ day. After that, the blood *β*-HCG and ultrasonography were reviewed every 5 days, and the uterus was cleared under the guidance of ultrasonography after the blood *β*-HCG was less than 10000 mIU/ml.

The observation group was treated with UACE combined with ultrasound-guided uterine curettage. UACE was performed, and lidocaine was used to locally anesthetize the right femoral artery area. After a successful percutaneous puncture of the right femoral artery, a 5F-uterine artery catheter was placed. Under digital subtraction angiography, guided by a coaxial guide wire, selective after intubation to the uterine artery, MTX (total dose of 50 mg/m^2^) was first perfused, and then gelatin sponge particles (> 560–710 *μ*m in diameter) were used to embolize the uterine artery. Ultrasound-guided uterine curettage was performed about 24 hours after embolization (Figures 1–4).

### 2.4. Observation Indicators

Clinical data of all patients were collected retrospectively (including the patient's age, cesarean section times, intraoperative blood loss, postoperative hospital stay, menstrual return to normal time, mass disappearance time, *β*-HCG recovery time, time from the last cesarean section, gestational week, diameter, thinnest muscle layer, CSP type, initial *β*-HCG level, uterine fibroids, fetal heartbeat, maximum gestational sac, and other data). The size of the cesarean section scar mass and *β*-HCG level were checked after the operation.

CSP classification: Type I: The thinnest part of the myometrium at the scar is more than 0.3 cm; Type II: The thinnest part of the myometrium at the scar is less than 0.3 cm but > 0.1 cm, and the fetal sac or mass is not protruding or slightly convex toward the bladder. Type III: The gestational sac was completely implanted in the myometrium at the site of the uterine scar and protruded outward toward the bladder, and the myometrium between the gestational sac and the bladder was markedly thinner, or even absent, with a thickness of ≤ 3 mm.

2 months postoperative efficacy evaluation criteria. Significant effect: the cesarean scar mass disappeared, and *β*-HCG returned to normal without complications. Effective: the cesarean section scar mass was decreased, and *β*-HCG gradually returned to normal, but the patient still had complications such as bleeding (> 200 ml). Invalid: The size of cesarean scar mass and *β*-HCG level did not change significantly. The patient had severe complications such as hemorrhage and uterine perforation and required laparotomy, laparoscopy, or vaginal surgery. Total effective rate = (Significant effect cases + Effective cases)/Total number of cases × 100%.

### 2.5. Statistical Methods

We used SPSS 22.0 software to process the data analysis, and measurement data were expressed as mean ± standard deviation ($\bar{x}$ ±*s*). Multigroup comparisons were performed using analysis of variance, and pairwise comparisons were performed using a *t*-test. Enumeration data were expressed as (%), and differences between groups were compared by the *χ*^2^ test. A logistic regression model was used for multivariate analysis. The test level was *α* = 0.05, and *P* < 0.05 indicates a statistically significant difference.

## 3. Results

### 3.1. UACE Angiography

### 3.2. Comparison of Postoperative Curative Effects between the Two Groups of Patients

After the operation, the total effective rate of patients in the observation group was 95.35%, which was higher than that of the control group (74.42%), and the difference was statistically significant (*P* < 0.05), as shown in Table 1.

### 3.3. Comparison of Intraoperative Bleeding and Postoperative Symptom Improvement Time between the Two Groups

After the operation, the volume of intraoperative blood loss, hospitalization period, menstrual recovery time, mass disappearance time, and *β*-HCG recovery time in the observation group were all lower than those in the control group, and the differences were statistically significant (*P* < 0.05), as shown in Table 2.

### 3.4. Univariate Analysis of Postoperative Efficacy in CSP Patients

Univariate analysis showed that the number of cesarean sections, gestational age, the maximum diameter of a gestational sac, the thinnest muscle layer, and the type of CSP could affect the postoperative curative effect of patients, and the differences were statistically significant (*P* < 0.05), as shown in Table 3.

### 3.5. Multivariate Analysis of Postoperative Curative Effects in CSP Patients

Multivariate Logistic analysis showed that gestational age, the maximum diameter of a gestational sac, the thinnest muscle layer, and the type of CSP were independent influencing factors of postoperative efficacy (*P* < 0.05), as shown in Tables 4-5.

## 4. Discussion

CSP refers to the implantation of a fertilized egg in the scar formed by the uterus after cesarean section, which is a special kind of ectopic pregnancy. At present, the etiology of CSP is still unclear, which may be related to endometrial injury or poor healing of uterine incision caused by surgical stimulation such as curettage and cesarean section [9, 10]. There was no significant difference in serum *β*-HCG concentration between cesarean section scar pregnancy patients and normal pregnancy, therefore, b-ultrasound is a commonly used method to check the CSP, and can also be used to evaluate the patient's postoperative recovery. The muscle layer at the cesarean section scar is weak and has poor contractility, and the gestational sac grows aggressively toward the blood vessel-rich muscle layer, which can easily damage the blood vessels and cause massive bleeding and even uterine rupture [11–13]. Therefore, early diagnosis and timely treatment of CSP are very important.

The results of this study showed that the total effective rate in the observation group was higher than that in the control group, and the intraoperative blood loss, postoperative hospital stay, menstrual recovery time, mass disappearance time, and *β*-HCG recovery time in the observation group were all lower than those in the control group. The reason is that UACE is an interventional therapy, and the risk of massive hemorrhage for patients is reduced by injecting an embolic agent into the uterine arteries. In addition, UACE combined with uterine curettage has many advantages, such as simple operation, promotion of patients' postoperative recovery, and maintenance of patients' fertility. This method of treatment can greatly improve the efficacy of the treatment of CSP, effectively improve the prognosis, and is an acceptable treatment method for patients [14, 15].

The results of this study showed that the number of cesarean sections, gestational age, the largest diameter of the gestational sac, the thinnest muscle layer, and the type of CSP could affect the postoperative efficacy of the patients. It is an independent factor affecting the postoperative efficacy of patients. The reason for this is that with the increase of gestational age, the pregnant uterus of patients with CSP gradually expanded, resulting in the reduction of muscle contraction force in the scar during cesarean section, and further leading to the occurrence of vaginal bleeding in patients, which affected the therapeutic effect of patients [16]. The maximum diameter of the patient's gestational sac increases, which leads to a more abundant blood supply around the gestational sac, which affects the effect of an intervention. The uterus also increases with the increase of the maximum diameter of the gestational sac, so that the contraction ability of the muscle layer at the cesarean section scar is further improved. It increases the risk of massive bleeding and uterine rupture, which is not conducive to the treatment of CSP patients [17, 18]. The thinner the thinnest muscle layer at the cesarean section scar, the lower the uterine contractility, and the easier it is for the gestational sac to penetrate the thinnest muscle layer of the uterine scar and enter the abdominal cavity when the muscle layer invasively grows, resulting in uterine rupture, which is not conducive to the patient's health and treatment efficacy [19, 20]. There are two types of CSP patients: endogenous type (CSP Type 1) and exogenous type (CSP Type 2). The gestational sac tissue of exogenous CSP patients grows aggressively toward the deep myometrium due to insufficient blood supply at the scar, which may cause a uterine rupture in the first trimester. Because the gestational sac in exophytic CSP patients invades and grows deep into the myometrium and is closely adhered to the uterus, the gestational sac is not easily separated from the uterus, and incomplete uterine curettage is prone to occur during uterine curettage [21, 22]. In addition, all patients have observed the development of their condition 6 months after treatment, no obvious adverse reactions were found in the treatment and postoperative follow-up of the two groups of patients in this study, indicating that UACE combined with curettage had high safety.

In conclusion, UACE combined with uterine curettage in the treatment of CSP can significantly improve the curative effect, reduce intraoperative bleeding, and improve the recovery time of postoperative-related symptoms. The gestational age, the largest diameter of the gestational sac, the thinnest muscle layer, and the type of CSP can independently affect the therapeutic effect of CSP patients. Fully understanding the high-risk factors affecting the efficacy of the treatment of CSP, timely preventive measures, and targeted nursing can effectively improve the prognosis and reduce the risk of CSP.

## Figures and Tables

**Figure 1:** The left uterine artery is slightly thickened, the spiral artery can be seen extending upward, and the uterine body is congested.

**Figure 2:** Complete embolization of left uterine artery.

**Figure 3:** The right uterine artery is slightly thickened, the spiral artery can be seen extending upward, and the uterine body is congested.

**Figure 4:** Right uterine artery completely embolized.

**Table 1:** Comparison of postoperative efficacy between the two groups of patients (*n*, %).

Group	Significant effect	Effective	Invalid	Total efficiency (%)
Control group (*n* = 43)	30	2	11	74.42 (32/43)
Observation group (*n* = 43)	38	3	2	95.35 (41/43)
*χ* ^*2*^ value				7.372
*P* Value				0.025

**Table 2:** Comparison of intraoperative bleeding and postoperative symptom improvement time between the two groups (*n*, $\bar{x}$ ±*s*).

Group	The volume of intraoperative blood loss (ml)	Hospitalization period (d)	Menstrual recovery time (d)	Mass disappearance time (d)	*β*-HCG recovery time (d)
Control group (*n* = 43)	66.42 ± 7.54	10.01 ± 4.55	40.02 ± 5.39	65.10 ± 8.45	60.35 ± 28.32
Observation group (*n* = 43)	39.26 ± 7.29	7.96 ± 1.32	36.96 ± 3.52	60.36 ± 6.11	46.88 ± 16.77
*t* value	16.982	2.837	3.117	2.981	2.684
*P* Value	0.000	0.006	0.003	0.004	0.009

**Table 3:** Univariate analysis of postoperative efficacy in patients with cesarean section scar pregnancy (*n*, %).

Influencing factors		Number of cases (*n* = 86)	Significant effect or effective (*n* = 73)	Invalid (*n* = 13)	*χ* ^*2*^ value	*P* Value
Age (year)	20∼30	39	36	3	3.065	0.080
	30∼40	47	37	10		
The number of cesarean sections (times)	≤1	54	50	4	5.653	0.017
	>1	32	23	9		
Time since last cesarean section (years)	≤5	39	31	8	1.620	0.203
	>5	47	42	5		
Gestational age (week)	≤8	48	45	3	6.655	0.010
	>8	38	28	10		
Maximum diameter of the gestational sac (cm)	≤3.6	61	55	6	4.560	0.033
	>3.6	25	18	7		
Thinnest muscle layer (cm)	≤0.21	36	27	9	4.714	0.030
	>0.21	50	46	4		
Type of CSP	Type 1	50	47	3	7.736	0.005
	Type 2	36	26	10		
Initial *β*-HCG (mIU/ml)	≤30000	37	33	4	0.938	0.333
	>30000	49	40	9		
Uterine fibroids	Yes	38	32	6	0.024	0.877
	No	48	41	7		

**Table 4:** Multifactor analysis assignment.

Influencing factors	Assignment
The number of cesarean sections	“≤1” = “0”; “>1” = “1”
Gestational age	“≤8” = “0”; “>8” = “1”
Maximum diameter of a gestational sac	“≤3.6” = “0”; “>3.6” = “1”
Thinnest muscle layer	“≤0.21” = “0”; “>0.21” = “1”
Type of CSP	“Type 1” = “0”; “type 2” = “1”

**Table 5:** Multivariate analysis of postoperative recovery in CSP patients (*n*, %).

Influencing factors	B	SE	Walds	Df	Sig	Exp (B)
The number of cesarean sections	0.811	0.601	1.821	1	0.177	2.250
Gestational age	0.474	0.241	3.885	1	0.049	0.622
Maximum diameter of a gestational sac	1.117	0.272	16.920	1	0.000	0.327
Thinnest muscle layer	0.553	0.242	4.830	1	0.028	1.704
Type of CSP	0.592	0.244	5.868	1	0.015	0.553

## Data Availability

The data can be obtained from the corresponding author upon reasonable request.
